The article "Application Development and Prospect of Family Therapy in China" was published in 2022. Journal: J Healthc Eng.

# Application Development and Prospect of Family Therapy in China

**DOI:** 10.1155/2022/4606101

**Published:** 2022-02-16

**Authors:** Feng Yao

**Affiliations:** Anhui Vocational College of Police Officers, Hefei 230031, China

## Abstract

Family therapy has been introduced into China for more than 30 years. This paper summarizes, reviews, reflects, and looks forward to the current research literature on family therapy in China from the aspects of methods, theories, and cultural adaptability. The conclusion is that family therapy that originated in the west has proved to be effective in China. Compared with the west, it is not sufficient in the research of family therapy in China. Further research can be done in the direction of cultural adaptability in two aspects in the future: first, clinicians need to strengthen their understanding of Chinese families; second, Chinese family therapy clinicians need to strengthen their case studies.

## 1. Introduction

Family therapy is a form of psychotherapy, and the theory came into existence in the 1970s and has since matured. Before that, psychotherapy focused on the improvement of individual personality and the settlement of inner conflicts. There were some blind spots when solving the whole family problems, because the family problems mainly resulted from the problems of family relations, interaction, boundaries, and rules. As a result, the family therapy was widely welcomed by the psychotherapists after it came into being. Family therapy was introduced into China in 1988 by the way of “Sino-German Psychotherapy Workshop.” After that, the techniques and methods of family therapy were transplanted in China, and the effectiveness and cultural adaptability were studied in clinical practice. Due to the prominent performance of family problems, youth education problems, and psychological problems in China in recent years, more and more psychotherapists, social workers, and psychological counselors from medical and nonmedical backgrounds are investing in the first line of family therapy and engaged in clinical practice. After years of practice, it has been found that there are many methodological and technical inadequacies in copying the western family therapy model. Therefore, timely review and summary of the current development of family therapy in China can better prospect the development of family therapy in China.

## 2. Literature Analysis

We conducted literature analysis on the current status of applied research of family therapy in China, including research methods, new progress, and relevant empirical studies. Advanced search was conducted on HowNet, using the title of “family therapy” as the article title. The time limit was from 2001 to 2021, and the total number of Chinese literature articles searched was 806. The research level distribution and topic distribution are shown in Tables 1 and 2.

The article "Application Development and Prospect of Family Therapy in China" was published in 2022. Journal: J Healthc Eng.

From the above distribution, the main research fields of home treatment in the past 20 years involve applied research, technology development, and clinical research, and the research topics mainly include theory of home treatment, effectiveness research of different models of home treatment, and clinical research. In the research field focusing on family therapy, the total number of articles related to “family therapy” and “culture” was 232 (accounting for 28.8%). In recent years, the number of articles discussing topics related to culture has shown an obvious upward trend (see Table 3).

Based on the above literature analysis, we mainly reviewed and analyzed the current research status of methods, theories, clinical applications, and cultural adaptability of family therapy in China and put forward suggestions on this basis.

## 3. Literature Review of the Application of Family Therapy in China

### 3.1. Introduction to Methods and Theories

Due to the differences in theoretical perspectives and clinical methods of traditional family therapy, there are many theoretical models for schism. Up till now, translations and published articles have also introduced various models of family therapy, among which systematic family therapy and structured family therapy are more introduced and introduced, followed by intergenerational family therapy and strategic family therapy.

For example, in the 16th issue of Jiangsu Education in 2020, the topic of systematic family therapy was specially opened to introduce systematic family therapy methods. Guo Jinmeng, Xing Chengju, etc. think that, with the enrichment and development of family therapy schools, the literature review on the field of family therapy for adolescents is carried out. Compared with the research status of family therapy abroad, there are different degrees of gaps in the research on the effectiveness of therapeutic intervention in practice, theory, and methods in China. It is of practical significance to review foreign research results and explore their development status in providing relevant practical evidence and promoting the development of adolescent family therapy in China [1]. It is worth noting that the Wai-Yung Lee team and the Zhao Xudong team have long carried out research in the domestic family treatment of training and research and promotion work. Hu Ziyi, Wai-Yung Lee, Wang Ailing, and others in 2006 published “On the concept of family treatment work” on the structure of family treatment introduced. Since 1988, Zhao Xudong and his team have also begun the introduction of the systemic family therapy model in China. Nine family dance series books such as “Personal Behavior from the Family System” written by Wai-Yung Lee were published in East China Normal University Press in 2019, while “Systemic Therapy and Counseling Text Book” translated by Zhao Xudong team was published by the Commercial Press in 2018. At the same time, Zhao Xudong team also translated or proofread the “Source of Heart” series such as “Manual on Systemic Psychotherapy” (2017), which had a certain influence in China.

The article "Application Development and Prospect of Family Therapy in China" was published in 2022. Journal: J Healthc Eng.

Some domestic scholars also introduced the new changes in family therapy under the influence of the new trend of thought in a timely manner. For example, Jiao Zhenghong and Zhao Xudong introduced five latest development trends of the influence of constructivism, feminism, and multiculturalism on family therapy in 2010. WANG Xin-jian and Lv Xiaokang (2007) also introduced that the family therapy with numerous schools originally presented an integrative trend in theory construction, skill level, and common factors contributing to curative effect. Zhao Fang (2010) also introduced the trend of integration of schools and technologies of contemporary family therapy, and these introductory articles provided researchers with timely understanding of the latest cutting edge of family therapy.

### 3.2. The Application of Research in Chinese Culture

Under the influence of philosophical hermeneutics, multiculturalism began to exert influence in western countries in the 1970s. It mainly advocated the recognition of cultural differences and emphasized the respect and equal coexistence among different cultures. The development of multiculturalism first spread to many fields of social science, and the field of psychology was also influenced by multiculturalism. For example, Szapocznik and Kurtines believe that although individuals are embedded in their own family context, each family unit is embedded in a context with “multiculturalism” (see Figure 1) [2]. Under the influence of the research on family therapy in the multicultural background, Chinese scholars have also carried out the research on the application and cultural adaptability of family therapy in Chinese culture.

#### 3.2.1. Application Effectiveness Study

For example, Zhao and Xu believed that the mental disorder patients and their family members who received family treatment had positive improvements at the individual and family levels through controlled study [3]. In addition, Zhao Xudong team also conducted an empirical study on systematic family treatment for anxiety disorder. Sim and Hu [4] reviewed and analyzed 39 articles on clinical empirical research of home treatment published in Chinese mainland journals from 1978 to 2006, and they showed that, compared with other psychological treatment modes, home treatment had obvious effects. During the 2020 epidemic, Chen Development and Zhao Xudong published research articles that supportive family system would play a buffer role against the pressure of social events in the epidemic process and conversely would amplify the destructive social pressure. Systemic family therapy technology could provide effective intervention to the epidemic psychological pressure of the public [5].

The article "Application Development and Prospect of Family Therapy in China" was published in 2022. Journal: J Healthc Eng.

However, a large number of studies on the effectiveness of family therapy in China have focused on the problematic behaviors, depression, and Internet addiction of teenagers, showing that domestic family therapy scholars mainly focus on the application of psychological problems of teenagers. For example, Xu Chaofan's doctoral dissertation carries out an empirical study on how family therapy interferes with families in problem of juvenile, and it concluded that family therapy can improve the family dynamics of problem of juvenile [6]. A domestic study conducted a controlled trial of adolescent depression patients, and the results showed that family treatment could alleviate the depressive symptoms of adolescents to a certain extent, improve the emotional state of their parents, and reduce family pressure [7]. Yao et al. explored the effect of structured family therapy on the improvement of depression among adolescents aged 13–18 years old through controlled trials. The results showed that the depression scores of the research groups receiving family therapy were significantly lower than those before treatment, and the effective rate reached 66%, indicating that structured family therapy had good effects on the improvement of depression among adolescents. Moreover, the improvement of family environment, such as the increase in the frequency of emotional expression among members, could effectively reduce the depression level of those with symptoms [8]. Combining social work case service, Kong Shiyi provided services for adolescent families taking drugs with structured family therapy, joint family therapy, and short-term strategic family therapy. The treatment results showed that structured family therapy adjusted the family structure, short-term strategic family therapy focused on family problems, and both had good effects in reshaping the family interaction model [9].

From the perspective of the study on the application effectiveness of family therapy, the application of family therapy in China is effective, and the application target is relatively concentrated on teenagers, which may also be related to the current situation of problematic families in China.

The article "Application Development and Prospect of Family Therapy in China" was published in 2022. Journal: J Healthc Eng.

#### 3.2.2. Applied Cultural Adaptability Research

After more than 30 years of clinical practice, some researchers have also found that there are some cultural conflict factors in family therapy originated from the West. For example, family therapists should pay attention to the values of the treated family and the cultural adaptability of family therapy in the application of Chinese family culture. Otherwise, the treatment relationship may be damaged, resulting in the failure of treatment. Although the family therapy that originated in the West cannot fully adapt to the Chinese family, the practice of family therapy in China shows that some basic ideas of family therapy such as the triangle relationship, alliance, family structure, and many theories of family dysfunction are also applicable to the Chinese family and have constructive significance. Therefore, the theory and technology of western family therapy in China's cultural adaptability research have important significance. As Taiwan Province has made a lot of achievements in the research of cultural adaptability in psychology in recent years, this part is mainly elaborated from two parts: Chinese mainland and Taiwan Province.

*(1) The Study of 3.2.2.1 Chinese Mainland.* In recent years, some psychologists and Chinese psychologists have carried out some research on the cultural adaptability of family therapy, and there are solutions to the current family problems. For example, Liu Liang's “Parents Do These 9 Things, Children Change from Weariness to Love” (2020) discusses the phenomenon that more children do not go to school in the current family therapy theoretically and practically. Yao Feng believed through research that the research on cultural adaptability of family therapy in China needs to be based on Chinese family ethics, which is a process of using family therapy technology to adjust the inappropriate ethical relationship and explore ethical resources [10]. Some studies also find that there are some differences in the findings and views of western family therapy in Chinese culture. For example, the empirical study of Zhao Xudong et al. has found that, for a more lasting effect, family therapists need to reflect on the cultural adaptability of family therapy in the application of Chinese culture. Another study of eating disorders found [11] that if the nuclear family relationship is too close, most patients do not feel good relationship between parents but feel excluded from the close relationship between parents; in this family structure, although the relationship between husband and wife is good, the function of the family structure is still out of balance, patients will feel parents two vertices is too close and will be excluded, and the structure of the core relationship between husband and wife in western families is different and also shows the cultural characteristics of family therapy.

The article "Application Development and Prospect of Family Therapy in China" was published in 2022. Journal: J Healthc Eng.

Although the existing literature on the study of cultural adaptability in a certain area was discussed, either standing in the context of western family therapy technology and theory to discuss the problems that need to be noticed in the application of family therapy in China or the family therapy technology directly to verify its effectiveness and put forward some reflective suggestions, cultural adaptability research is not deep enough. Liang Zhixiu, Sun Dan, and others believe that the Chinese family's emphasis on authority and hierarchy of the characteristics of the structured family therapy in China's application provides a basis for agreement; although it discusses some issues of cultural conflict, it did not go deep into the Chinese cultural framework to explore the root causes of the conflict and how to solve the conflict specific countermeasures. However, the research on cultural adaptability in the context of Chinese family culture is almost blank.

*(2) A Study of the Taiwan Province Region in 3.2.2.2, China.* Psychotherapy research in Taiwan Province, China, is mainly focused on the local fit of the study, mainly representative of several psychologists such as Yang Guoshu's local fit criteria, Huang Guangguo's psychology of containing the perturbation culture, Song Wenli's Chinese cultural psychology, Yu Dehui phenomenological orientation of local clinical psychology, and Li Weilun's psychological suffering and ethical relations.

The first is the theory of yang guoshu. In 1993 and 2005, Yang Guoshu published his localization research results with the theme of “Chinese native psychology” in Studies of Native Psychology and Chinese Native Psychology respectively. In his 2005 article, Yang Guoshu replaced “indigenous psychology” with “indigenous psychology” as the exact name to describe the psychological research of non-Western psychologists rooted in the local cultural society. In this article, Yang Guoshu tries to construct the localization psychology status that is the psychology development “time/history” and “space/region” two axial. In contrast to the self-questioning imposition-style research strategy formed by applying the concept of western psychology to non-Western people, Yang Guoshu believes that the native psychologists must consciously use thematic or quasithematic research strategies. The focus of this research strategy is to return to the local history, culture, and social context, which can be “to reincorporate the local history, culture, and social factors into their research.” In addition, Yang Guoshu also proposed the concepts of “cultural fit” and “local fit” [12–15].

The article "Application Development and Prospect of Family Therapy in China" was published in 2022. Journal: J Healthc Eng.

The second is Huang Guangguo's theory. Huang Guangguo believes [16] that if the local psychologists adhere to the positivist research orientation, without being clearly aware of the phenomenon/ontology dualism in the epistemology of limitations, he will not only take the hermeneutic orientation of the researchers on the knowledge of conflict and opposition [17], but his research may also be because of bias to collect empirical data that appear trivial and difficult to understand. On the contrary, if we adopt the research orientation of postpositivism, deeply think about the cultural value and action wisdom behind each kind of social action, and devote ourselves to construct the theory that can not only reflect the common mind of human beings, but also explain the mentality of people in the local society, we can break the barrier between empirical science and hermeneutics. In Habermas's book Knowledge and Human Purport, knowledge is divided into three different sciences [18]. The microworld of science to be constructed by local psychology should contain three different sciences, which can meet the three different “cognitive interests” of human beings: the science of experience-analysis; history-the science of interpretation; and critical science. Huang Guangguo's “native psychological framework” has two characteristics: (1) using postpositivism realism in western philosophy of science as epistemology, and getting the position of dialogue with western psychological theory. (2) With the cultural psychologist Richard Shweder's assertion of “one mind, multiple mindsets” as the basis and “Confucian relativism” as the connotation of Chinese culture, the universal “self-mandala model” and the theoretical model of “human feelings and face” are constructed to counteract the Western psychological theory. Huang Guangguo proposed the universalism psychology theory based on the Confucian relativism to counter the western individualism psychology as its cultural strategy of native psychology. Huang Guangguo thinks first of all to positivism as his native psychological basis; secondly, it is necessary to establish a psychological theory of containing the culture of taking care, which is his “self-mandala model” and “human feelings and face” two theoretical models based on Confucian relativism; finally, to debate and dialogue on theoretical issues with western psychologists, in action to implement the “theoretical competition, to contend with” the doctrine of strategy [19, 20].

The article "Application Development and Prospect of Family Therapy in China" was published in 2022. Journal: J Healthc Eng.

Again, Song Wenli think local psychology is put forward by Taiwan Province psychologists to western psychology as “the other”; that is to say, the other is the speaker. However, when Taiwan Province's psychologists want to use their own language to say their own psychological experience, they found themselves in a state of “aphasia” [21, 22].

Fourthly, Yu Dehui believes that those who need to pay attention to local psychology “in suffering” are also “in language” and “in culture,” “People in the cultural language construction of local culture of self-perception, at the same time, people also use cultural language to place others” disease body position. The position of the sick is socially constructed—the relationship and treatment that the vulnerable sick will be placed in are all in the context of cultural history. Yu Dehui went on to point out that the most significant thing in Chinese life is the interpersonal order, and the core of life's misery is the interpersonal disorder, such as the antagonism between the depressed patients and their relatives, the fragmentation of the life of the trauma patients, and the entanglement of human ethics. Yu Dehui and Li Weilun believe that the ethical collapse of these phenomena is not that there is no ethics, but that the ethical order in which life was originally based can no longer be relied on, forming a “black hole of ethics” or a state of “ethics is not good enough.” Therefore, Yu Dehui puts forward the understanding that “suffering is always ethical suffering” and thus advocates for ethical therapy as the starting point for the construction of the localization of clinical psychology [23, 24].

Summing up the localization of the above four scholars, we can see that the four scholars' arguments point to the life experience as a cultural life is the basis for the reconceptualization of the theory. In summary, the localization goal of Yang Guoshu and Huang Guangguo is to establish the local psychological theoretical knowledge based on the regional culture, which makes Chinese psychology possess the theoretical subjectivity different from that of western psychology. However, Song Wenli and Yu Dehui hold the view that life subjectivity should be taken as the basis, because all kinds of experiences in contemporary life are the basis for the reconceptualization of western theories and traditional viewpoints. Thus, after reobserving the discourses of the four scholars, we find that the goal of the native psychological strategy with theoretical subjectivity and life subjectivity is not to arrive at “separation” but to arrive at “communication.” The concepts of “local fit” and “cultural fit” by Mr. Yang Guoshu, the research on the relationship between psychotherapy and ethics by Yu Dehui, Li Weilun, and others, and the views of Song Arts and Science and Huang Guangguo all put forward the basic ideas and principles of psychotherapy localization. They all go deep into the ontology of Chinese culture and strive to carry out psychotherapy based on the “understanding” of Chinese culture. The family culture in Taiwan Province region and the family culture in the mainland have a high degree of homogeneity, so the research in Taiwan Province region needs our high attention.

The article "Application Development and Prospect of Family Therapy in China" was published in 2022. Journal: J Healthc Eng.

## 4. Conclusion and Discussion

Based on the above review of research articles on family therapy in China, the author puts forward the following reflections and prospects for the application and research of family therapy in China.

### 4.1. The Application of Family Therapy in China Is Generally Effective, but the Research Is Not Deep Enough

At present, clinical and empirical studies in China have proved that family therapy that originated from the West is also effective in China. Particularly, there are many studies on the therapeutic effects of adolescent problems and psychosomatic disorders, which also reflect the prominent practical needs of contemporary family problems and adolescent mental health problems in China. However, there are still some shortcomings. In the current situation, compared with the western research, the family therapy research in China is not enough.

A recent study outside China used the quasiexperimental design method to measure the effectiveness of structured strategic family therapy in adolescent families with mental health problems [25]. The experiment lasted for 10 years, and the results were compared before and after the experiment. It was found that structured strategic family therapy played a promoting role in reducing adolescent psychological problems, improving parents' competence and recovering family functions. Compared with the family therapy in China, there are few long-span studies, and some effects need to be verified over a long period of time. Case study and introduction are not deep enough, and long-term observation is not enough. This is also an aspect that needs to be improved in family treatment in China in the future.

In addition, at the level of methods and technologies, although there are many translations and introductions of the related methods and technologies of western family therapy in China, overall, the advantages and methods of various schools have not been integrated at the theoretical level. The schools of family therapy have not high degree of differentiation and have more in common. The next step needs to be the induction and integration of different school theories. At the application level, there are many related studies due to the prominent manifestations of adolescents' nonattendance at school, suicide, and various psychosomatic disorders in family problems in China in recent years. However, some domestic family therapists have weak consciousness of problems and insufficient reflection on reality, so the research is not enough. At the level of research methods, the qualitative research methods are not fully applied, and the quantitative research lacks in-depth follow-up study. At the level of research objects, from the literature, the current domestic research on the efficacy of family therapy focuses too much on adolescents, and the articles on the localization of family therapy and cultural adaptability are not deep enough.

The article "Application Development and Prospect of Family Therapy in China" was published in 2022. Journal: J Healthc Eng.

### 4.2. The Future Can Be In-Depth Study in the Direction of Cultural Adaptability from Two Aspects

Facing the future, we think that the research of family therapy in China should pay attention to the adaptability research in Chinese culture, go deep into the family culture context, find the way to “understand” the Chinese family, find a breakthrough on this basis, and use the family therapy theory and technology to solve family problems. Zhao Xudong made several recommendations regarding the development of family therapy in China: first, a long-term follow-up study of the population receiving family therapy and a study of the longer-term efficacy of family therapy; second, professionals from different industries can participate in the family therapy study together to reach cross-disciplinary conclusions; third, attention should be paid to scientific research methods, as well as the process of family therapy [26]. Attention should also be paid to the impact of family therapy in different cultural environments, actively developing family therapy with local cultural adaptability [27]. Liu Dan, a systematic family therapist, recalled that his inner understanding when receiving the systematic family therapy training was a process of gradually understanding the family therapy under the Chinese culture: “When I followed Simon's guidance and returned to my own culture, savored it carefully and pondered it slowly, I found that the thinking and life of the Chinese people were systematic. Only the systematic features exist in the Chinese unconscious. Few have studied and applied it clearly, clearly and scientifically. When I constantly try to use Chinese characters, history, stories, architecture and other different forms as the medium to transmit, the system view and system-based consulting technology becomes easy to understand, be mastered, and be applied” [28]. Therefore, we believe that “understanding” of family history and culture should be strengthened, and solid clinical research work should be carried out in the process of case treatment to carry out family treatment in the context of Chinese culture.

4.2.1 From the philosophical hermeneutics sense, in the Chinese culture of psychology research, first of all, we need to understand the contemporary people's psychological experience and feelings, in the context of the traditional understanding of the current problem, which requires a modern interpretation of the traditional context, after the interpretation to build a new meaning and widen the new understanding. Therefore, it is necessary to do relevant research in the context or coordinate system of the local culture. Only in this way can the research be realistic. In the research method, to achieve “understanding,” it does not need to predict and control the problem as the center, as long as we can solve the problem, and we can be flexible to use a variety of methods [29]. When we use the concept of “context,” we are trying to understand a person's psychological distress and problem behavior from two dimensions of the current relationship and the context of historical development, and to find a solution from the system context, which is also the thinking that family therapists need to have, that is, “system thinking.” Systematic thinking makes the ways to assist a person to change more diversified and no longer limited to individuals [30].

The article "Application Development and Prospect of Family Therapy in China" was published in 2022. Journal: J Healthc Eng.

Researchers of family therapy in China need to strengthen their “understanding” of Chinese families. If the family therapist does not develop cultural sensitivity, it is difficult to “understand” the problem family. And the new transformation of family culture on the basis of “understanding” may transform the seemingly “problem” factors into the positive factors of Chinese family growth. Treatment can only be carried out on the basis of understanding, which also needs to be carried out within a time development context, which requires a modern interpretation of the development context of Chinese family history, building a new meaning and adding a new understanding after the interpretation. Therefore, it is necessary to do relevant research in the context or coordinate system of the local culture. Only in this way can the research be realistic. In terms of research methods, it is also necessary to achieve “understanding,” rather than just prediction and control, focusing on problems. As long as problems are solved, various methods can be flexibly applied [29].

Regarding the understanding of Chinese family in the western family therapy theory and technology, we think we should pay attention to the following three issues: first, what is the current research progress of family therapy in China? Second, is family therapy effective in China and what are the cultural conflicts? Thirdly, how can family therapy be applied in the context of Chinese family culture? To address these three issues, we suggest that we first need to be familiar with the current status of theoretical research on family therapy in China and abroad, such as the latest research on family function and family resilience in family therapy. On this basis, we should focus on the latest research on the cultural adaptability of family therapy in Chinese families and also pay attention to the research in Taiwan Province area with high cultural homogeneity, so as to identify problems, and then propose problems and find solutions in the research on the development context of Chinese culture and the two-way interaction of family therapy. It is shown in Figure 2.

4.2.2 Family therapy clinical workers in China need to strengthen case studies. Qualitative research such as case studies, field investigations, and grounded theory tends to focus on people's understanding and experience of the world rather than looking for causal relationships, describing and giving possible explanations for events and experiences, rather than predicting. Qualitative research is to investigate people who are in their own life field (i.e., in naturally occurring scenarios such as families, schools, hospitals, etc.), which are open systems, in which many factors continuously develop and interact with each other [31]. However, family therapy pays more attention to the reduction of the life field and the situation and context, so it is more suitable for qualitative research. Due to the multicultural characteristics of family therapy, it requires that Chinese family therapists should be culturally sensitive, able to accurately analyze and judge the cultural background and cultural values of the family encountered in the clinical process, and make targeted adjustments to the theory and technology of family therapy.

The article "Application Development and Prospect of Family Therapy in China" was published in 2022. Journal: J Healthc Eng.

In Figure 3, we propose to find research clues from the existing theories, verify the clinical application of cases in Chinese family culture, identify problems and propose assumptions at the level of cultural adaptability, and further verify the case treatment process and propose a new theoretical model suitable for Chinese families, so as to gradually construct a case study route with its own cultural characteristics of family treatment mode.

In this model, in the case study, we need to put forward theoretical assumptions and selection methods and talk with them under the framework of family therapy. However, the samples we choose and the treatment process need to be culturally sensitive. At the same time, the analysis of the treatment process should be carried out in the context of Chinese family culture. Finally, the previous theories are revised to form new theoretical assumptions as shown in Figure 3. It is also worth noting that, due to the lack of long-term research on family therapy case studies in China, the depth and time span of case studies need to be strengthened to make up for the insufficient depth of family therapy case studies.

## Figures and Tables

**Figure 1:** Analysis model of individuals and families embedded in multicultural environment.

**Figure 2:** Family therapy “understanding” the thinking diagram of Chinese families.

**Figure 3:** Route of case study.

**Table 1:** Study level distribution (data source from CNKI).

Fields	Application research	Technology development	Clinical research	Business research	Policy research	The development of research	Engineering research
The percentage	42.8	28.6	13	3.1	2.5	2.5	1.9

**Table 2:** Distribution of main topics (data source from CNKI).

Fields	Family therapy	Structured family therapy	Family therapy model	Systematic family therapy	Schizophrenia	Satya family therapy	Schizophrenic patients	Treatment and care
The percentage	60.1	8.2	6.8	9.7	4.5	4.2	4	2.5

**Table 3:** Trends in publication of topics related to culture and family therapy (data source from CNKI).

Year	2002	2004	2006	2008	2010	2012	2014	2016	2018	2020
Number of articles	4	4	9	4	6	15	10	12	24	20

## Data Availability

The datasets used and/or analyzed during the current study are available from the corresponding author upon reasonable request.
